The article "In Silico and In Vitro Screening Constituents of Eclipta alba Leaf Extract to Reveal Antimicrobial Potential" was published in 2022. Journal: Evid Based Complement Alternat Med.

# In Silico and In Vitro Screening Constituents of *Eclipta alba* Leaf Extract to Reveal Antimicrobial Potential

**DOI:** 10.1155/2022/3290790

**Published:** 2022-08-17

**Authors:** Rahul Kumar Sharma, Shabana Bibi, Hitesh Chopra, Muhammad Saad Khan, Navidha Aggarwal, Inderbir Singh, Syed Umair Ahmad, Mohammad Mehedi Hasan, Mahmoud Moustafa, Mohammed Al-Shehri, Abdulaziz Alshehri, Atul Kabra

**Affiliations:** ^1^Department of Pharmacology, Amar Shaheed Baba Ajit Singh Jujhar Singh Memorial College of Pharmacy, Bela, Punjab, India; ^2^Department of Biosciences, ShifaTameer-e-Millat University, Islamabad, Pakistan; ^3^Yunnan Herbal Laboratory, College of Ecology and Environmental Sciences, Yunnan University, Kunming 650091, China; ^4^Chitkara College of Pharmacy, Chitkara University, Rajpura 140401, Punjab, India; ^5^Department of Biosciences, Faculty of Sciences, COMSATS University Islamabad, Sahiwal, Pakistan; ^6^Maharishi Markandeshwar College of Pharmacy, Maharishi Markandeshwar, Mullana, Ambala 133207, Haryana, India; ^7^Department of Pharmaceutical Sciences, Guru Jambheshwar University of Science and Technology, Hisar 125001, Haryana, India; ^8^Department of Bioinformatics, Hazara University Mansehra, KPK, Pakistan; ^9^Department of Biochemistry and Molecular Biology, Faculty of Life Science, Mawlana Bhashani Science and Technology University, Tangail 1902, Bangladesh; ^10^Department of Biology, College of Science, King Khalid University, 9004 Abha, Saudi Arabia; ^11^Department of Botany and Microbiology, Faculty of Science, South Valley University, Qena, Egypt; ^12^King Khalid University, College of Medicine, Abha, Saudi Arabia; ^13^University Institute of Pharma Sciences, Chandigarh University, Gharuan, 140413 Mohali, Punjab, India

## Abstract

Phytochemicals have been shown to possess multiple bioactives and have been reported to showcase many medicinal effects. A similar kind of evaluation of phytoconstituents for their antimicrobial action has been reported, based on in vitro and in silico data. The goal of the research was to explore bioactive phytoconstituents of *Eclipta alba* leaf for antimicrobial activity. The antimicrobial activity was validated by both molecular docking and antimicrobial assay. Bioactive metabolites were identified using GC-MS. The antimicrobial and antimycobacterial activity of *Eclipta alba* leaves was investigated using the Kirby–Bauer well diffusion method and the rapid culture—MGIT™ DST method against a variety of human pathogens, as well as *Mycobacterium tubercu*losis (H37Rv) and *Mycobacterium tuberculosis* bacteria resistant to isoniazid and rifampicin. *Eclipta alba's* GC-MS studies confirmed the detection of 17 bioactive constituents. The extract demonstrates the highest antibacterial activity against *Escherichia coli* (sensitive), *Pseudomonas aeruginosa* (sensitive) and methicillin-resistant *Staphylococcus aureus* (MRSA), and *Pseudomonas aeruginosa* susceptible and MRSA (sensitive) with zone of inhibition of 27 mm, 24 mm, and 32 mm respectively. The extract showed no effect on *Mycobacterium tuberculosis* (H37Rv) and *Mycobacterium tuberculosis* bacteria resistant to isoniazid and rifampicin in antimycobacterial activity testing. Molecular docking investigation revealed that three compounds (phthalic acid, isobutyl octadecyl ester, hexadecanoic acid, 1(hydroxymethyl)1,2-ethanediylester, and 2,myristynoyl pantetheine) have generated the best results in terms of binding energies and significant interactions with key residues of target protein 3-hydroxydecanoyl-acyl carrier protein dehydratase (FabA) and confirm its activity as antimicrobial inhibitors. These two-dimensional plots show significant protein-ligand binding interactions (van der Waals interactions, hydrogen bond, alkyl, and Pi-alkyl interactions). ADMET (absorption, distribution, metabolism, excretion, and toxicity) results additionally support the drug-likeness characteristics of concluded potential compounds. The experimental and computational results demonstrated that methanolic extract of *Eclipta alba* leaves had antimicrobial effects for specific infections due to the presence of phytochemical compounds.

## 1. Introduction

A diverse diversity of critters, microscopic organisms, and species call the world home. Microbes are minute creatures that may be found in almost every environment, from deep seas to heated places such as geysers and even volcanoes [1]. Bacteria ranging from gram negative to gram positive, as well as fungi and viruses, make up these microscopic forms of life. Bacteria are microscopic organisms that are thought to be among the first forms of life on earth, surviving even in the most extreme temperatures, such as those found in the earth's crust. *Escherichia coli, Klebsiella pneumoniae, Pseudomonas aeruginosa, Staphylococcus aureus, Mycobacterium tuberculosis, Aspergillus fumigatus, and Candida albicans* are one of the most deadly microorganisms. Microbial infection occurs when pathogens or microorganisms infect healthy human cells, turning them sick. Antibiotics such as penicillin, cephalosporin, tetracycline, aminoglycosides, and others are used to treat a variety of microbiological infections. The antibiotics work by having multiple targets that include (i) cell wall synthesis, (ii) protein biosynthesis, (iii) cell membrane destruction, (iv) DNA replication and repair, and (v) metabolic inhibition. However, the most important issue that develops during antibiotic treatment is antimicrobial resistance, which has raised serious concerns about microbial infections. Almost every microbe develops resistance to infections. These resistant microorganisms are difficult to treat, resulting in catastrophic illnesses that kill millions of people around the world. The growth in antimicrobial resistance is mostly due to antibiotic prescribing and distribution practices in developing nations. Antimicrobial resistance is responsible for more than 7 lakh fatalities worldwide. Antimicrobial resistance will kill 350 million people by 2050, according to a report done by the World Health Organization (WHO) [2]. Antimicrobial resistance is expected to have a particularly negative impact on developing countries. As antimicrobial resistance has expanded fast, antibiotic treatments have become less effective and, in some cases, ineffective.

Herbs and medicinal plants provide a wealth of primary and secondary metabolites, including carbohydrates, proteins, lipids, alkaloids, glycosides, tannins, and a variety of other compounds [3–11]. Traditional medicine has historically relied on herbs and plants. Herbs are thought to be a treasure trove of phytochemicals with a diverse variety of biological activities [6, 8, 11–14]. The herbs that house these various elements are a natural gift. Alkaloids, flavonoids, and saponin are some of the secondary metabolites that have significant therapeutic value. Multiple chronic diseases, such as diabetes, cardiovascular disease, chronic fatigue syndrome, and a variety of infections, are treated as a result of the existence of such metabolites. Many scientific research studies have shown that these primary and secondary metabolites have the ability to treat a variety of acute and chronic disorders. These metabolites safeguard the human body by inhibiting harmful microorganisms that cause infectious diseases in one or more ways.

Antibiotic resistance is becoming more common in the modern world. As a result, alternative methods for the treatment of infectious disorders are required [15–17]. Due to their diverse biological and therapeutic activity, large safety margins, and cheaper prices, herbal medicines are in considerable demand as a source of basic health care in both developed and developing nations. Herbal metabolites, which occur in the protoplasm of the plant cell in a mixed or pooled form of more than one molecule, are harmless and would overcome disease resistance [10, 11]. *Eclipta alba* is commonly known as Bhringaraja belonging to the Asteraceae family. The whole plant parts are used as hepatoprotective [18], immunomodulatory [19], anti-inflammatory and analgesic [20, 21], hair growth and alopecia [22], antidepressant [23], antidiabetic [24], and nervine tonic [25, 26]. The aim of this study was to find out chemical constituents of methanolic extract of *Eclipta alba* that reveals antimicrobial activity.

## 2. Materials and Methods

### 2.1. Material and Preparation of Extract

Plant material of *Eclipta alba* leaves was collected from a nursery of the adjacent Rajasthan University in Jaipur (26.8853°N, 75.8208°E). The duplicate specimen was authenticated in the Department of Botany, Rajasthan University, Jaipur, for species identification. The dried powder of the leaves (25 gm) was extracted with 150 ml 80 percent methanol using a Soxhlet apparatus for 24 hours and then filtered through a 0.45 m filter membrane. In a rotator evaporator, the filtrate was evaporated in reduced pressure and dried at 55°C [27].

### 2.2. GC-MS Analysis

For the GC-MS analysis, an Agilent system with a mass spectrometer detector and split injection system was used. A HP5MS capillary column was installed in the GC (30m × 250m; film thickness: 0.25 m). The injector temperature is 280°C, the initial oven temperature is 50°C, and then it progressively increased to 300°C at 25°C/min and kept for 10 minutes, according to the temperature manual. At a pressure of 17.69 psi and a flow rate of 2.1 ml/min, helium was used as the carrier gas. The samples were dissolved in methanol, and a 1 l aliquot was automatically injected. The WILEY and NIST (National Institute of Standards and Technology) libraries for botanical chemicals were used to identify the MS of separated components. GC-MS detection of phytoconstituents of methanolic extract of *Eclipta alba* was based on the computer evaluation of mass spectra of samples through comparison of peaks and retention time.

### 2.3. Determination of Antimicrobial Activities

Kirby–Bauer well diffusion and MGIT™ DST methods were used to determine antimicrobial activity of methanolic extract of *Eclipta alba* at CIRD (Centre for Innovation, Research & Development) from Dr. B. Lal Institute of Biotechnology and Research Centre, Jaipur, Rajasthan.

#### 2.3.1. Bacterium Is Chosen for Study

Bacterium was chosen for antimicrobial evaluation using two separate sets (sensitive and resistant) for gram positive, gram negative, and mycobacterium. *Candida albicans* and *Aspergillus fumigates* were chosen for antifungal testing. The Microbial Culture Collection Division (MCRD) of CIRD provided all of the pure microbial cultures used in this investigation:1—*Escherichia coli* (sensitive), ATCC 25922; 2—*Escherichia coli* (ESBL), ATCC 35218; 3—*Klebsiella pneumoniae* (sensitive), MTCC 3384; 4—*Klebsiella pneumonia* (ESBL), ATCC 7000603; 5—*Staphylococcus aureus* (sensitive), ATCC 25923; 6—*Staphylococcus aureus* (MRSA), ATCC 4330; 7—*Pseudomonas aeruginosa* (sensitive), ATCC27853; 8—*Pseudomonas aeruginosa* (resistant) clinical isolate—CIRD-MCRD; 9—*Mycobacterium tuberculosis* H37Rv; 10—*Mycobacterium tuberculosis* clinical isolate—CIRD-MCRD; 11—*Candida albicans* clinical isolate—CIRD-MCRD; and 12—*Aspergillus fumigatus* clinical isolate—CIRD-MCRD.

#### 2.3.2. Sample Processing

From the stock solution, two strengths of the methanolic extract of *Eclipta alba* leaves were made (100 mg/ml and 200 mg/ml), and then, the dilution series for the compound was prepared, with 50 *µ*l utilized in each well. Positive controls for antibacterial and antifungal activities were streptomycin and itraconazole (5 mg/ml concentration).

#### 2.3.3. Agar Plates Were Prepared for the Antibacterial Activity

The susceptibility test media that have been validated by CLSI (Clinical & Laboratory Standards Institute) for screening antimicrobial activity by disk/well diffusion susceptibility testing are the Mueller–Hinton agar medium and the Sabouraud dextrose agar medium.

#### 2.3.4. Preparation of Inoculum

*Escherichia coli, Klebsiella pneumoniae, Staphylococcus aureus, Pseudomonas aeruginosa, and Candida* cultures were inoculated in peptone water and incubated for 30 minutes at 37°C, whereas Aspergillus cultures were inoculated in normal saline and incubated for 48 hours at 28°C.

#### 2.3.5. Inoculum Size of Bacteria Was Adjusted Using McFarland Turbidity Standard as Reference

The bacterial suspensions were compared to 0.5 McFarland Turbidity Standard.

#### 2.3.6. Swabbing of the Liquid Cultures

Swabs of Candida and Aspergillus cultures were placed on the Sabouraud dextrose agar surface, whereas bacterial cultures were placed on the Mueller–Hinton agar surface.

#### 2.3.7. Loading Test Solutions into the Wells

In the wells, 50 *µ*l of stock dilutions (100 mg/ml and 200 mg/ml of *Eclipta alba* methanolic extract) was poured.

#### 2.3.8. Incubation

The bacterial and Candida plates were kept at 37°C for 24 hours, whereas the Aspergillus plates were kept at 28°C for 7 days.

### 2.4. Antimycobacterial Susceptibility Testing

The antimycobacterial activity of *Eclipta alba* methanolic extract was assessed by automated antibacterial susceptibility testing against (1) *Mycobacterium tuberculosis* (H37Rv) and (2) *Mycobacterium tuberculosis* bacteria resistant to isoniazid and rifampicin, both using the MGIT™ DST method (Mycobacteria Growth Indicator Tube).

The extract of *Eclipta alba* was diluted to the 10 mg/ml concentrations. A total of seven MGITs were labeled, and 0.8 ml supplement was added to each tube. 1st tube was then kept aside, and extract of 100 *μ*l from the stock of 100 mg/ml was added to the respective tubes. Tubes were mixed properly and kept aside. 1 : 100 dilution of DST inoculum (*Mycobacterium tuberculosis* (H37Rv)) was prepared for the growth control tube (1st tube), and 1 : 5 dilution of DST inoculum (*Mycobacterium tuberculosis* (H37Rv) and *Mycobacterium tuberculosis* (MDR)) was prepared for tubes. 0.5 ml of 1 : 100 dilution was added to the 1st tube (growth control tube). 0.5 ml of 1 : 5 dilution was added to other respective tubes. All tubes were incubated in MGIT-320 instrument at 370 C.

### 2.5. Computational Analysis

#### 2.5.1. Construction of Chemical Compound Database

There is literature accessible that emphasizes the necessity of identifying prospective antimicrobial treatments, as well as the fact that currently available synthetic drugs are not particularly healthy due to various severe side effects [28, 29]. The identification of novel medications for various ailments is greatly facilitated by computer-aided screening applications [18, 19]. A database of 17 compounds was used, and an integrated computer-aided technique implies to identify innovative drugs to combat antimicrobial disease. The structures of each chemical drug were created using ChemDraw software, and the information from each structure was cross-checked against the PubChem database (Figure 1) to avoid ambiguity before being saved in SDF format for further investigation [30].

#### 2.5.2. Enzyme/Target Protein Structure Selection for Docking Studies

In the research of antimicrobial disease, understanding the disease mechanism and then selecting an appropriate protein structure to begin the drug design pipeline are essential, as it can explain the critical parameters required to clarify the action of bound ligands, which are drugs that can selectively inhibit the activity of the 3-hydroxydecanoyl-acyl carrier protein dehydratase (FabA) [20, 21]. Therefore, the FabA protein (PDB ID : 4B0C) structure was chosen to perform this study including molecular docking experiment, which was conducted to investigate protein-ligand binding interactions between the two molecules, protein and selected drug [31].

#### 2.5.3. Molecular Docking and Interaction Analysis

To comprehend the protein-ligand bonded configuration and explain the molecular mechanism of small drug-like entities involved in cellular pathways, molecular docking is the most relevant technique [32]. An ESI-LCMS identified 17 compounds for molecular docking, and a three-dimensional (3D) structure of the FabA protein (PBD ID : 4B0C) in PDB format was imported into the MOE software for molecular docking analysis [33]. Heteroatoms, three-dimensional protonation, and water molecules were removed from the protein structure to prepare it for the docking approach, as well as the default ligand attached to the target protein. Based on previous literature [34], an active site in the selected protein (4B0C) is identified, and structural optimization is carried out using the following parameters: the addition of hydrogen atoms, energy minimization using the Amber14 force field method with chiral constraints, and geometrical parameters. The surfaces and maps panel module allows for the adjustment of the transparency of the front and backward surfaces, which results in the display of significant residues in the selected substrate binding site of the 4B0C protein in its native conformation, by the use of the surfaces and maps panel module [34]. The MOE software creates a database of 17 compounds identified through experimental investigation, which is then saved with the MDB extension for future study. This database is used to run molecular docking simulations. After refinement, the top-ranked poses (postures) were subjected to the calculation of binding free energies (G), which were then evaluated using the scoring function (GBVI/WSA dg) [35]. It was discovered that the number of chemical contacts (interactions) may be used to create a valid scoring scheme that results in a docking score for the correct binding postures such as hydrogen, Pi, and van der Waals interactions [36]. To better understand how FabA inhibitors interact with the target protein's chosen pocket, the MOE database containing the docked complex was rigorously displayed in Figure 2.

#### 2.5.4. In Silico Pharmacokinetic/ADMET Profile Calculations

The best compound was determined based on docking outcomes to estimate the ADMET (absorption, distribution, metabolism, excretion, and toxicity) profile, which is a crucial parameter for the drug-like screening of chemical compounds [37]. For ADMET profile estimation, Swiss ADME [38] and DataWarrior tools were used [39].

## 3. Results

### 3.1. GC-MS Profiling of Extract of *Eclipta alba*

Table 1 displays findings of GC-MS profiling of *Eclipta alba* leaves, which revealed the presence of 17 main phytoconstituents such as n-Undecane, cyclohexasiloxane-dodecamethyl, nonahexacontanoic acid, 2,4-ditertbutylphenol, 1,2-benzenedicarboxylic acid-butyl octyl ester, 2-myristynoyl pantetheine, palmitic acid methyl ester, phthalic acid-butyl nonyl ester, phthalic acid, isobutyl octadecyl ester, phen-1-4-diol,2,3-dimethyl-5-trifluoromethyl, 10-octadecenal,butyl-9,12-octadecadienoate, 13-octadecenoic acid methyl ester, methyl stearate, hexadecanoic acid, 1(hydroxymethyl)1,2-ethanediylester, hexasiloxane, 1,1,3,3,5,5,7,7,9,9,11,11-dodecamethyl, and sitosterol in Table 1, and Figure 1 shows the GC-MS chromatogram of a methanolic extract of *Eclipta Alba* leaves, as well as the mass spectra of the various phytoconstituents detected.

#### 3.1.1. Antimicrobial Activity of *Eclipta alba*

The antimicrobial activity was measured using the Kirby–Bauer well diffusion method, which yielded a zone of inhibition as a result. Streptomycin (5 mg/ml) and itraconazole (5 mg/ml) were the reference drug used as a positive control for test organisms.  Table 2 shows the antibacterial activity of the methanolic extract of *Eclipta alba*, which is depicted in Figures 3–5. The result of the study showed that a methanolic extract of *Eclipta alba* had an inhibitory effect on the test organisms in both concentrations. The extract showed antibacterial activity against *Pseudomonas aeruginosa* (sensitive) (100 mg/ml-26 mm, 200 mg/ml-27 mm), *Staphylococcus aureus* (MRSA) (100 mg/ml-23 mm, 200 mg/ml-24 mm), and *Pseudomonas aeruginosa* (sensitive) (100 mg/ml-29 mm, 200 mg/ml-32 mm). However, against *E. coli* (sensitive and ESBL), *Klebsiella pneumoniae* (sensitive and ESBL), *Pseudomonas aeruginosa* (resistant), *Candida albicans*, and *Aspergillus fumigates*, the extract had no antibacterial activity. The crude extract showed the highest antimicrobial activity against *Pseudomonas aeruginosa* (sensitive). *Eclipta alba* leaves possess significant antimicrobial activity as assessed from different zones of inhibitions observed during the study and confirm their inhibitory effect over the growth of tested pathogens; however, the antimicrobial activity is concentration-dependent. Both 100 mg/ml and 200 mg/ml showed antimicrobial activity for selective pathogens.

### 3.2. Antimycobacterial Activity of *Eclipta alba* Leaves

The antimycobacterial activity of methanolic extract of *Eclipta alba* at 100 mg/ml did not inhibit the development of *Mycobacterium tuberculosis* (H37Rv) or *Mycobacterium tuberculosis* (MDR) isolate at concentration of 0.1 mg/vial, as shown in Table 3.

### 3.3. Computational Analysis

#### 3.3.1. Molecular Docking and Interaction Analysis

The 3-hydroxydecanoyl-acyl carrier protein dehydratase (FabA) (PDB ID : 4B0C) structure has been utilized. For the purpose of molecular docking and interaction research, a biomolecule structure lacking bound ligands and with a substantial active site was created [34] (Figure 6). The database includes 17 bioactive compounds discovered by ESI-LCMS and submitted to MOE with MDB extension and protein-ligand docking simulations in the active site of FabA using the dock module of MOE program [33]. To control microbe-created illness, phytochemicals with the best binding positions and molecular interactions with the most important amino acids comprise the mechanism of inhibition of FabA. By evaluating the identified active binding site, residues with substantial activity were highlighted.  Table 4 lists the dock score and RMSD values determined by MOE program for the database of 17 compounds with FabA protein. While the three compounds with the highest dock scores have been shown to have the best binding poses, and substantial binding interactions with active site residues of the target FabA protein are within a range of 4.5 Å, Figure 7 and Table 4 provide a detailed view of the best docking results.

All three selected potential hits have van der Waals, hydrogen bonds, alkyl, and Pi-alkyl bonding, and the majority of the selected active site is hydrophobic in nature (Table 5). The dock score range is between −7.3511 and −6.9875 Kcal/mol, indicating that these hits have been confined to the optimal conformation within the target protein's selected active site (Figures 2, 8, and 9).

#### 3.3.2. In Silico Pharmacokinetic/ADMET Profile Calculations

With the advancements in bioinformatic data and tools, it is feasible to compute the pharmacokinetic (ADMET) and drug-like characteristics to screen the highly significant drug from a huge dataset with a reduced likelihood of rejection during the first phase of drug development [40]. Previous medical literature has addressed *in silico* pharmacokinetics and toxicity estimates [41, 42]. In this investigation, the physiochemical descriptors and drug-likeness of three key isolated phytochemicals with docking findings were used to estimate the ADMET characteristics using the drug design and discovery, and Web-based Swiss ADME and Osiris molecular property explorer have been employed. In Table 6, these three phytochemicals exhibited relatively acceptable ADMET property values.

Although it is critical to understand the status of a chemical or drug, it is possible that the predicted pharmacokinetic properties of selected phytochemicals are insufficient to understand the membrane permeability of selected phytochemicals. This is due to the fact that some phytochemicals are poorly metabolized by the body, while others are well metabolized, because the high log P and molecular weight values of phytochemicals and sometimes could not fulfill the drug-like filtration rules, while most important is the Lipinski rule [43] of drug-likeness that is acceptable in the case of selected one phytochemical, 2,myristynoyl pantetheine, and other two phytochemicals, phthalic acid, isobutyl octadecyl ester and hexadecanoic acid,1(hydroxymethyl)1,2-ethanediylester, results show minor violation in this study.

However, the most important cytochrome P450 isoforms (CYP1A2, CYP2C19, CYP2C9, CYP2D6, and CYP3A4) have been explained by the calculation. This calculation is demanding for isoforms of the cytochrome P450 superfamily in the metabolism and elimination of substances from the liver, and their mechanism investigations [44]. As a result of medication administration, inhibitors of cytochrome P45 stimulate phytochemical interactions that may not be able to be utilized in metabolism and may be stored as harmful material in the body. These pharmacokinetic values for three phytochemicals are not very excellent, and as a result, they have an impact on the bioavailability of medications. The lipophilicity of selected phytochemicals is also important in the bioavailability of these compounds. Because several drug-like parameters involved in the oral administration of drugs are being violated, poor lipophilic compounds are associated with poor gastrointestinal (GI) absorption and have low BBB permeability, and it is critical to understand the receptor and drug interactions involved in the diseases of the central nervous system [45]. Phytochemicals with low solubility, such as those listed in Table 7, help to explain absorption and distribution since they have a low level of solubility.

It was determined that pan-assay interference compounds (PAINS) and Brenk calculations were the chemical defects in a selected medication/chemical that needed to be addressed before moving forward with the initial step of drug development [46, 47]. In this study, three chosen phytochemicals were shown to exhibit modest PAINS and Brenk unwanted medicinal warnings, as well as certain molecularly damaging moieties, which might provide prerequisite information for the modification of chemical structure prior to proceeding into the development phase. While the toxicity estimation by Osiris molecular property explorer [48] demonstrated that all two phytochemicals are tending towards the safe results in terms of mutagenic, tumorigenic, irritant, and reproductive effects, one compound phthalic acid, isobutyl octadecyl ester seems to be toxic and subsequently drug-likeness and drug scores were estimated on the basis of cumulative ADMET parameters as shown in Table 6.

## 4. Discussion

India has wide plant diversity. Plants are rich sources of secondary metabolites that exhibit various biological activities. In present time, the scope of plant-based study has been increased. Some of the phytoconstituents are already proven as antimicrobial agents. Phytoconstituents such as coumarin, flavonoids, phenolics, alkaloids, terpenoids, tannins, and polyacetylenes have been shown to have bacteriostatic, bactericidal, and fungicidal effects against a variety of human pathogens in multiple studies [49, 50]. Some of the other research studies also supported that inhibitory activity of secondary metabolites is attributed by interfering biochemical pathway, protein synthesis, and decay of outer membrane [51–53]. The goal of this study was to determine the phytoconstituents and antibacterial and antimycobacterial activity of *Eclipta alba* leaf methanolic extract. The result of GC-MS showed seventeen compounds that have various biological activities. The methanolic extract of *Eclipta alba* was found to have antimicrobial action against *E. coli* (sensitive), *Pseudomonas aeruginosa* (sensitive), *Staphylococcus aureus* (MRSA), and *Pseudomonas aeruginosa* (sensitive) at both doses, with the highest impact at 200 mg/ml. The antimycobacterial activity of the extract revealed that it was able to grow *M. tuberculosis* (H37Rv) and *M. tuberculosis* (MDR). It is observed that, during the study, antimicrobial activity of extract exhibited higher zone of inhibition than standard drug against *Pseudomonas aeruginosa* (sensitive) at 200 mg/ml. Molecular docking results were interpreted by MOE, and they presented remarkable binding energies in Kcal/mol and binding interactions in terms of van der Waals, hydrogen bond, alkyl, and Pi-alkyl interactions and hence proved that highlighted three potential hits (phthalic acid, isobutyl octadecyl ester, hexadecanoic acid,1(hydroxymethyl)1,2-ethanediylester, and 2,myristynoyl pantetheine) have been bounded in the best conformation within target protein selected active site (Figure 4). Hydrogen bonds are very important for the stability of docked complex; therefore, phthalic acid, isobutyl octadecyl ester has generated three hydrogen bonds with PHE114 and ARG152 residues, while CYS80, LEU83, VAL111, and ILE154 residues have been involved in in the alkyl and Pi-alkyl binding interactions (Figure 2). Hexadecanoic acid,1(hydroxymethyl)1,2-ethanediylester has generated one hydrogen bond with GLY115 residue, and PHE71 and PHE113 residues are associated with Pi-alkyl interaction (Figure 8). 2,Myristynoyl pantetheine has presented three hydrogen bonds with CYS80, PHE113, and GLY115 residues, while LEU83, TRP87, LEU118, ALA121, VAL149 residues have been involved in the alkyl and Pi-alkyl bond formation to make the docked complex stable conformation (Figure 9). In silico ADMET results showed that all three selected hits exhibited moderately acceptable properties as enlisted in Tables 6 and 7, and these significant predictions could be helpful in the further improvement and optimization of these chemicals in the early stages of drug development phase.

## 5. Conclusion

This study found that a methanolic extract of *Eclipta alba* leaves has antibacterial activity against a small number of human diseases, but not all of them. By the computational drug design and discovery pipeline, three potential hits were screened: phthalic acid, isobutyl octadecyl ester, hexadecanoic acid,1((hydroxymethyl)1,2-ethanediylester, and 2,myristynoyl pantetheine, and they presented the best and stable conformation within active site of target 3-hydroxydecanoyl-acyl carrier protein dehydratase (FabA); further studies are needed for the development of plant investigated to modify to certain dosage forms, that can be used for management of infections and can be further taken for clinical evaluation.

## Figures and Tables

**Figure 1:** GC-MS chromatogram of methanolic extract of *Eclipta alba.*

**Figure 2:** Graphical representation of molecular docked complex of phthalic acid, isobutyl octadecyl ester in the vicinity of active binding site of alpha-glucosidase protein, best bounded pose of phthalic acid, isobutyl octadecyl ester presenting the potential of hydrogen bonding capacity (green represents hydrogen bond acceptor region, and purple represents the hydrogen bond donor region) with active binding site residues (a), and two-dimensional plot presenting binding interactions of the phthalic acid and isobutyl octadecyl ester with target alpha-glucosidase protein (b).

**Figure 3:** Antimicrobial activity plates of methanolic extract of *Eclipta alba* leaves. (a) Extract concentration of 100 mg/ml. (b) Extract concentration of 200 mg/ml.

**Figure 4:** Antimicrobial activity plates of methanolic extract of *Eclipta alba* leaves. (a) Extract concentration of 100 mg/ml. (b) Extract concentration of 200 mg/ml.

**Figure 5:** Antimicrobial activity plates of methanolic extract of *Eclipta alba* leaves. (a) Extract concentration of 100 mg/ml. (b) Extract concentration of 200 mg/ml.

**Figure 6:** Two-dimensional representation of selected 17 compounds used for molecular docking analysis.

**Figure 7:** Selected active binding site of the 3-hydroxydecanoyl-acyl carrier protein dehydratase (FabA) for molecular docking investigation.

**Figure 8:** Graphical representation of molecular docked complex of hexadecanoic acid,1(hydroxymethyl)1,2-ethanediylester in the vicinity of active binding site of alpha-glucosidase protein, best bounded pose of hexadecanoic acid,1(hydroxymethyl)1,2-ethanediylester presenting the potential of hydrogen bonding capacity (green represents hydrogen bond acceptor region, and purple represents the hydrogen bond donor region) with active binding site residues (a), and two-dimensional plot presenting binding interactions of the hexadecanoic acid,1(hydroxymethyl)1,2-ethanediylester with target alpha-glucosidase protein (b).

**Figure 9:** Graphical representation of molecular docked complex of 2,myristynoylpantetheine in the vicinity of active binding site of alpha-glucosidase protein, best bounded pose of 2,myristynoylpantetheine presenting the potential of hydrogen bonding capacity (green represents hydrogen bond acceptor region, and purple represents the hydrogen bond donor region) with active binding site residues (a), and two-dimensional plot presenting binding interactions of the 2,myristynoylpantetheine with target alpha-glucosidase protein (b).

**Table 1:** GC-MS analysis of *Eclipta alba* leaf methanolic extract.

RT	Peak area	Peak height	% Area	Mol. Wt.	Formula	Compound name
12.87	186648902.6	34060302.71	21.34	156	C_11_H_24_	n-Undecane
18.77	6899331.8	1400651.25	0.79	444	C_12_H_36_O_6_Si_6_	Cyclohexasiloxane, dodecamethyl
23.83	7103149.34	1599701.7	0.81	998	C_69_H_138_O_2_	Nonahexacontanoic acid
24.34	74602969.17	23151534.73	8.53	206	C_14_H_22_O	2,4-Ditertbutylphenol
31.8	9882056.21	3020324.92	1.13	334	C_20_H_30_O_4_	1,2-Benzenedicarboxylic acid, butyl octyl ester
32.75	11665954.16	2084631.75	1.33	484	C_25_H_44_N_2_O_5_S	2,Myristynoyl pantetheine
33.16	126428686.5	43947724.68	14.45	270	C_17_H_34_O_2_	Palmitic acid, methyl ester
33.68	27993487.97	8476191.01	3.2	334	C_20_H_30_O_4_	Phthalic acid, butyl nonyl ester
34	10431119.98	3241088.3	1.19	474	C_30_H_50_O_4_	Phthalic acid, isobutyl octadecyl ester
35.32	7229742.55	2058149.86	0.83	206	C_9_H_9_F_3_O_2_	Phen-1,4-diol,2,3-dimethyl-5-trifluoromethyl
35.88	6592001.96	2283063.28	0.75	266	C_18_H_34_O	10-Octadecenal
36	12643029.67	4970293.44	1.45	336	C_22_H_40_O_2_	Butyl-9,12-octadecadienoate
36.12	35963115.18	11345325.23	4.11	296	C_19_H_36_O_2_	13-Octadecenoic acid, methyl ester
36.51	68288303.2	24209016.08	7.81	298	C_19_H_38_O_2_	Methyl stearate
42.09	11856463.62	3940854.12	1.36	568	C_35_H_68_O_5_	Hexadecanoic acid,1(hydroxymethyl)1,2-ethanediylester
44.44	6083348.57	1301181.23	0.7	430	C_12_H_38_O_5_Si_6_	Hexasiloxane,1,1,3,3,5,5,7,7,9,9,11,11-dodecamethyl
45.01	196695067.6	24458173.31	22.48	414	C_29_H_50_O	Sitosterol

**Table 2:** Antimicrobial activities of *Eclipta alba* leaves.

Name of microorganism	Zone of inhibition (mm)		
	Extract (MEEA)		Streptomycin and itraconazole conc.—5 mg/ml
	Conc.—100 mg/ml	Conc.—200 mg/ml	
*E. coli (sensitive)*	—	—	29 mm
*E. coli (ESBL)*	—	—	22 mm
*Klebsiella pneumoniae (sensitive)*	—	—	20 mm
*Klebsiella pneumonia (ESBL)*	—	—	19 mm
*Staphylococcus aureus (sensitive)*	26 mm	27 mm	27 mm
*Staphylococcus aureus (MRSA)*	23 mm	24 mm	25 mm
*Pseudomonas aeruginosa (sensitive)*	29 mm	32 mm	27 mm
*Pseudomonas aeruginosa (resistant)*	—	—	21 mm
*Candida albicans*	—	—	26 mm
*Aspergillus fumigatus*	—	—	17 mm

**Table 3:** Antimycobacterial activity of *Eclipta alba* leaves.

Tube#	Compound name	Extract	Concentration	Growth reported *Mycobacterium tuberculosis* (H37Rv)	Growth reported *Mycobacterium tuberculosis* (MDR)
1	Positive control	Nil	Nil	Yes	Yes
2	Negative control 1 (NTC-1)	Methanol	100 *µ*l methanol	Yes	Yes
3	*Eclipta alba*	Extract	100 *µ*l (volume) from the stock of 10 mg/ml	Yes	Yes

**Table 4:** Dock score and RMSD values calculated for the database of 17 compounds with 3-hydroxydecanoyl-acyl carrier protein dehydratase (FabA).

Compound name	PubChem ID	Dock score	RMSD	Compound name	PubChem ID	Dock score	RMSD
n-Undecane	14257	−4.6636	1.8191	10-Octadecenal	5365012	−5.716	1.3214
Cyclohexasiloxane, dodecamethyl	10911	−5.8971	1.0899	Butyl-9,12-octadecadienoate	102296	−5.8145	2.0079
Nonahexacontanoic acid	590850	−3.5110	1.1000	13-Octadecenoic acid, methyl ester	5364506	−5.7048	2.3566
2,4-Ditertbutylphenol	7311	−4.6286	1.6918	Methyl stearate	8201	−5.6709	1.5301
1,2-Benzenedicarboxylic acid, butyl octyl ester	66540	−5.7232	1.4823	Hexadecanoic acid,1(hydroxymethyl)1,2-ethanediylester	99931	−7.3152	2.2839
2,Myristynoyl pantetheine	535560	−6.9806	1.4732	Hexasiloxane, 1,1,3,3,5,5,7,7,9,9,11,11-dodecamethyl	71338303	−6.8487	2.8723
Palmitic acid, methyl ester	8181	−5.6478	1.4231	Sitosterol	222284	−5.344	1.2484
Phthalic acid, butyl nonyl ester	6786	−5.5100	1.1786	Butyl-9,12-octadecadienoate	102296	−5.8145	2.0079
Phthalic acid, isobutyl octadecyl ester	6423451	−7.3511	1.9858				

**Table 5:** Summary of molecular docking results of top 3 dock score hits with 3-hydroxydecanoyl-acyl carrier protein dehydratase (FabA).

Chemical#	Compound names	Dock score (Kcal/mol)	Functional residues	Binding interactions
Hit-1	Phthalic acid, isobutyl octadecyl ester	−7.3511	GLY79, CYS80, LEU83, TRP87, GLY107, SER108, VAL111, PHE114, GLY115, GLN116, VAL149, ARG152, Ile154, TYR155	Van der Waals, hydrogen bond, alkyl, Pi-alkyl

Hit-2	Hexadecanoic acid,1(hydroxymethyl)1,2-ethanediylester	−7.3152	PHE71, GLU72, GLY73, ASP74, GLY79, CYS80, LEU83, TRP87, PHE113, GLY115, GLN116, LEU118, ARG152, GLU153, TYR155	Van der Waals, hydrogen bond, Pi-alkyl

Hit-3	2,Myristynoyl pantetheine	−6.9806	GLY79, CYS80, LEU83, TRP87, VAL111, PHE113, PHE114, GLY115, GLN116, VAL117, LEU118, THR120, ALA121, VAL149, ARG152, ILE154, TYR155	Van der Waals, hydrogen bond, alkyl, Pi-alkyl

**Table 6:** ADMET profile of selected three phytochemicals calculated by Osiris molecular property explorer.

Chemical descriptors	Phthalic acid, isobutyl octadecyl ester	Hexadecanoic acid,1(hydroxymethyl)1,2-ethanediylester	2,Myristynoyl pantetheine
Irritant	Toxic effects	No effects	No effects
Mutagenic	Toxic effects	No effects	No effects
Tumorigenic	Toxic effects	No effects	No effects
Reproductive properties	Toxic effects	No effects	No effects
cLogP	10.24	12.25	3.95
Solubility	−725	−8.22	−5.4
MW	474.0	568.0	484.0
TPSA	52.6	72.83	141.0
Drug-likeness	−30.1	−26.0	−43.1
Drug score	0.20	0.08	0.24

**Table 7:** Pharmacokinetic and drug-like profile of selected three phytochemicals estimated by Swiss ADME server.

Chemical parameters	Phthalic acid, isobutyl octadecyl ester	Hexadecanoic acid,1(hydroxymethyl)1,2-ethanediylester	2,Myristynoyl pantetheine
Molecular weight (MW) (g/mol)	474.72	568.91	484.69
Rotatable bonds	23	34	21
Hydrogen bond acceptors (HBAs)	4	5	5
Hydrogen bond donors (HBDs)	0	1	4
Molar refractivity (MR)	145.14	174.09	136.31
Total polar surface area (TPSA) (Å)	52.60	72.83	141.03
LogPo/w (iLOGP)	6.03	8.17	4.53
LogS (ESOL)	−7.83	−9.97	−4.86
Solubility (mg/mL)	7.05*e* – 06	6.12*e* + 08	6.67*e* − 03
Class	Poorly soluble	Poorly soluble	Poorly soluble
GI absorption	Low	Low	Low
BBB permeant	No	No	No
P-gp substrate	No	Yes	Yes
CYP1A2 inhibitor	No	No	Yes
CYP2C19			
Inhibitor	No	No	Yes
CYP2C9 inhibitor	No	No	No
CYP2D6 inhibitor	No	No	No
CYP3A4 inhibitor	No	No	No
Log Kp (skin permeation) (cm/s)	1.95	0.20	-5.42
Lipinski	1 violation		
MLOGP > 4.15	2 violations		
MW > 500, MLOGP > 4.15	No violations		
Veber	No violations	No violations	Violations, TPSA > 140
Bioavailability score	0.55	0.17	0.85
PAINS	No alert	No alert	No alert
Brenk	1 alert		
More_more_2_esters	1 alert		
More_more_2_esters	2 alerts		
Thioester, triple_bond			
Synthetic accessibility	4.14	5.91	5.36

## Data Availability

The data used to support the findings of the study can be from the corresponding author upon request.

## References

[1] Bansal H., Singla R. K., Behzad S., Chopra H., Grewal A. S., Shen B. (2021). Unleashing the potential of microbial natural products in drug discovery: focusing on streptomyces as antimicrobials goldmine. *Current Topics in Medicinal Chemistry*.

[2] (2019). *No Time to Wait: Securing the Future from Drug-Resistant Infections Report to the Secretary-General of the United Nations *.

[3] Chopra H., Bibi S., Singh I. (2022). Green metallic nanoparticles: biosynthesis to applications. *Frontiers in Bioengineering and Biotechnology*.

[4] Khalil M. S., Shakeel M., Gulfam N. (2022). Fabrication of silver nanoparticles from ziziphus nummularia fruit extract: effect on hair growth rate and activity against selected bacterial and fungal strains. *Journal of Nanomaterials*.

[5] Saleem S., Bibi S., Yousafi Q. (2022). Identification of effective and nonpromiscuous antidiabetic drug molecules from penicillium species. *Evidence-based Complementary and Alternative Medicine*.

[6] Singh Bakshi I., Chopra H., Sharma M., Kaushik D., Pahwa R., Haryanto (2022). Herbal bioactives for wound healing application. *Herbal Bioactive-Based Drug Delivery Systems*.

[7] Singla R. K., Behzad S., Khan J. (2022). Natural kinase inhibitors for the treatment and management of endometrial/uterine cancer: preclinical to clinical studies. *Frontiers in Pharmacology*.

[8] Bhattacharya T., Soares G. A. B. E., Chopra H. (2022). Applications of phyto-nanotechnology for the treatment of neurodegenerative disorders. *Materials*.

[9] Walia V., Kaushik D., Mittal V. (2022). Delineation of neuroprotective effects and possible benefits of AntioxidantsTherapy for the treatment of alzheimer’s diseases by targeting mitochondrial-derived reactive oxygen species: bench to bedside. *Molecular Neurobiology*.

[10] Chopra H., Mishra A. K., Baig A. A., Mohanta T. K., Mohanta Y. K., Baek K. H. (2021). Narrative review: bioactive potential of various mushrooms as the treasure of versatile therapeutic natural product. *Journal of Fungi*.

[11] Chopra H., Dey P. S., Das D. (2021). Curcumin nanoparticles as promising therapeutic agents for drug targets. *Molecules*.

[12] Chopra H., Bibi S., Kumar S., Khan M. S., Kumar P., Singh I. (2022). Preparation and evaluation of chitosan/PVA based hydrogel films loaded with honey for wound healing application. *Gels*.

[13] Chopra H., Bibi S., Islam F. (2022). Emerging Trends in the Delivery of Resveratrol by Nanostructures: Applications of Nanotechnology in Life Sciences. *Journal of Nanomaterials*.

[14] Kour J., Chopra H., Bukhari S. (2022). Nutraceutical-A deep and profound concept. *Nutraceuticals and Health Care*.

[15] Islam F., Bibi S., Meem A. F. K. (2021). Natural bioactive molecules: an alternative approach to the treatment and control of COVID-19. *International Journal of Molecular Sciences*.

[16] Biswas P., Hasan M. M., Dey D. (2021). Candidate Antiviral Drugs for COVID-19 and Their Environmental Implications: A Comprehensive Analysis. *Environmental Science and Pollution Research International*.

[17] Bibi S., Wang Y.-B., Tang D.-X., Kamal M. A., Yu H. (2020). Prospects for discovering the secondary metabolites of cordyceps sensu lato by the integrated strategy. *Medicinal Chemistry*.

[18] Rangineni V., Sharada D., Saxena S. (2007). Diuretic, hypotensive, and hypocholesterolemic effects of Eclipta alba in mild hypertensive subjects: a pilot study. *Journal of Medicinal Food*.

[19] Jayathirtha M. G., Mishra S. H. (2004). Preliminary immunomodulatory activities of methanol extracts of Eclipta alba and *Centella asiatica*. *Phytomedicine*.

[20] Udayashankar A. C., Nandhini M., Rajini S. B., Prakash H. S. (2019). Pharmacological significance of medicinal herb eclipta alba L.-A review. *International Journal of Pharmaceutical Sciences and Research*.

[21] Leal L. K. A. M., Ferreira A. A. G., Bezerra G. A., Matos F. J. A., Viana G. S. B. (2000). Antinociceptive, anti-inflammatory and bronchodilator activities of Brazilian medicinal plants containing coumarin: a comparative study. *Journal of Ethnopharmacology*.

[22] Datta K., Singh A. T., Mukherjee A., Bhat B., Ramesh B., Burman A. C. (2009). Eclipta alba extract with potential for hair growth promoting activity. *Journal of Ethnopharmacology*.

[23] Mishra S., Jena M., Pal A. (2013). Evaluation of antidepressant activity of Eclipta alba using animal models. *Asian Journal of Pharmaceutical and Clinical Research*.

[24] Ananthi J., Prakasam A., Pugalendi K. V. (2003). Antihyperglycemic activity of Eclipta alba leaf on alloxan-induced diabetic rats. *The Yale Journal of Biology Medicine*.

[25] Vaidya A. D. B. (1997). The Status and Scope of Indian Medicinal Plants Acting on Central Nervous System. *Indian Journal of Pharmacology*.

[26] Thakur V. D., Mengi S. A. (2005). Neuropharmacological profile of Eclipta alba (linn.) hassk. *Journal of Ethnopharmacology*.

[27] Simões M., Bennett R. N., Rosa E. A. S. (2009). Understanding Antimicrobial Activities of Phytochemicals against Multidrug Resistant Bacteria and Biofilms. *Natural Product Reports*.

[28] Tapsell L. C., Hemphill I., Cobiac L. (2006). Health Benefits of Herbs and Spices: The Past, the Present, the Future. *The Medical Journal of Australia*.

[29] Lai P., Roy J. (2004). Antimicrobial and chemopreventive properties of herbs and spices. *Current Medicinal Chemistry*.

[30] Rampone S., Pagliarulo C., Marena C. (2020). In silico analysis of the antimicrobial activity of phytochemicals: towards a technological breakthrough. *Computer Methods and Programs in Biomedicine*.

[31] Orlando B. J., Malkowski M. G. (2016). Crystal structure of rofecoxib bound to human cyclooxygenase-2. *Acta Crystallographica Section F Structural Biology Communications*.

[32] Shah M., Rahman H., Khan A. (2022). Identification of *α*-glucosidase inhibitors from scutellaria edelbergii: ESI-LC-MS and computational approach. *Molecules*.

[33] Vilar S., Cozza G., Moro S. (2008). Medicinal chemistry and the molecular operating environment (MOE): application of QSAR and molecular docking to drug discovery. *Current Topics in Medicinal Chemistry*.

[34] Moynié L., Leckie S. M., McMahon S. A. (2013). Structural insights into the mechanism and inhibition of the *β*-hydroxydecanoyl-acyl carrier protein dehydratase from *Pseudomonas aeruginosa*. *Journal of Molecular Biology*.

[35] Aldeghi M., Heifetz A., Bodkin M. J., Knapp S., Biggin P. C. (2016). Accurate calculation of the absolute free energy of binding for drug molecules. *Chemical Science*.

[36] Ahmad S., Ranaghan K. E., Azam S. S. (2019). Combating tigecycline resistant Acinetobacter baumannii: a leap forward towards multi-epitope based vaccine discovery. *European Journal of Pharmaceutical Sciences*.

[37] Khan M. S., Mehmood B., Yousafi Q. (2021). Molecular docking studies reveal rhein from rhubarb (rheum rhabarbarum) as a putative inhibitor of ATP-binding cassette super-family G member 2. *Medicinal Chemistry*.

[38] Daina A., Michielin O., Zoete V. (2014). ILOGP: a simple, robust, and efficient description of n-octanol/water partition coefficient for drug design using the GB/SA approach. *Journal of Chemical Information and Modeling*.

[39] Sander T., Freyss J., Von Korff M., Rufener C. (2015). DataWarrior: an open-source program for chemistry aware data visualization and analysis. *Journal of Chemical Information and Modeling*.

[40] Zeb M. A., Rahman T. U., Sajid M. (2021). GC-MS analysis and in silico approaches of Indigofera heterantha root oil chemical constituents. *Compounds*.

[41] Saleem U., Shehzad A., Shah S. (2021). Antiparkinsonian activity of Cucurbita pepo seeds along with possible underlying mechanism. *Metabolic Brain Disease*.

[42] Saleem U., Bibi S., Shah M. A. (2021). Anti-Parkinson’s evaluation of Brassica juncea leaf extract and underlying mechanism of its phytochemicals. *Frontiers in Bioscience*.

[43] Tian S., Wang J., Li Y., Li D., Xu L., Hou T. (2015). The Application of in Silico Drug-Likeness Predictions in Pharmaceutical Research. *Advanced Drug Delivery Reviews*.

[44] Donato M. T., Castell J. V. (2003). Strategies and Molecular Probes to Investigate the Role of Cytochrome P450 in Drug Metabolism: Focus on in Vitro Studies. *Clinical Pharmacokinetics*.

[45] Pajouhesh H., Lenz G. R. (2005). Medicinal chemical properties of successful central nervous system drugs. *NeuroRx*.

[46] Mok N. Y., Maxe S., Brenk R. (2013). Locating sweet spots for screening hits and evaluating pan-assay interference filters from the performance analysis of two lead-like libraries. *Journal of Chemical Information and Modeling*.

[47] Pouliot M., Jeanmart S. (2016). Pan Assay Interference Compounds (PAINS) and Other Promiscuous Compounds in Antifungal Research. *Journal of Medical Chemistry*.

[48] Nalini C. N., Raga Deepthi S., Ramalakshmi N., Uma G. (2011). Toxicity risk assesment of Isatins. *Rasayan Journal of Chemistry*.

[49] Thomas E., Aneesh T. P., Thomas D. G., Anandan R. (2013). GC-MS analysis of phytochemical compounds present in the rhizomes of Nervilia aragoana GAUD. *Asian Journal of Pharmaceutical and Clinical Research*.

[50] Motaleb M. A. (2011). *Selected Medicinal Plants of Chittagong Hill Tracts*.

[51] Dholaria M., Desai P. (2018). Antibacterial and phytochemical studies with cytotoxicity assay of kalanchoe pinnata leave extract against multi-drug resistant human pathogens isolated from UTI. *International Journal of Pharmaceutical Sciences and Research*.

[52] Shriram V., Khare T., Bhagwat R., Shukla R., Kumar V. (2018). Inhibiting bacterial drug efflux pumps via phyto-therapeutics to combat threatening antimicrobial resistance. *Frontiers in Microbiology*.

[53] Ellington M. J., Ganner M., Warner M., Cookson B. D., Kearns A. M. (2009). Polyclonal multiply antibiotic-resistant methicillin-resistant *Staphylococcus aureus* with Panton-Valentine leucocidin in England. *Journal of Antimicrobial Chemotherapy*.

